The article "Effect of Traditional Chinese Medicine on Allergic Rhinitis in Children under Data Mining" was retracted in 2023. Reasons: unreliable results or conclusions; lack of ethics approval or compliance; concerns about the data; concerns about the peer review.

# Effect of Traditional Chinese Medicine on Allergic Rhinitis in Children under Data Mining

**DOI:** 10.1155/2022/7007370

**Published:** 2022-06-01

**Authors:** Min Shen, Jianghai Liu, Kuanhong Wang

**Affiliations:** Department of Paediatrics, Zhejiang Putuo Hospital, Zhoushan, 316100 Zhejiang, China

## Abstract

The data mining analysis of the medication rule and the curative effect of traditional Chinese medicine in treating allergic rhinitis in children was performed by using the association rule Apriori algorithm. The model of interest degree was introduced to improve the Apriori algorithm, and the performance difference of the algorithm before and after improvement was analyzed. Traditional Chinese medicine prescriptions for the treatment of allergic rhinitis in children were selected from the dictionary of Chinese medicine formulations. The frequency, frequent itemsets, and the improved Apriori algorithm of each prescription were analyzed comprehensively. The results showed that both the execution time of the improved Apriori algorithm and the number of mining association rules were signally lower. 102 Chinese herbal compounds were selected, in which the occurrence frequency of Flos magnoliae was the highest (67 times, 5.33%). The occurrence frequency of diaphoretic drugs was the highest (412 times, 32.78%) in drug types. The occurrence frequency of Yu Ping Feng powder was the highest (21 times, 20.59%) in the Chinese herbal compound. After the association rule analysis of the improved Apriori algorithm, Perilla frutescens, Saposhnikovia divaricata, ginseng, Notopterygium root, and Astragalus propinquus Schischkin were often mixed with liquorice, and Flos magnoliae were usually mixed with Fructus xanthii and black plum. Compared with the conditions before treatment, the sign scores of children with allergic rhinitis were remarkably decreased after treatment with traditional Chinese medicine compounds (*P* < 0.05). The mining performance of the Apriori algorithm was improved by introducing an interest-based model. The treatment of traditional Chinese medicine on allergic rhinitis in children was combined with children's physiological and pathological characteristics of children, which used mild medicines.

## 1. Introduction

Allergic rhinitis in children mainly refers to noninfectious inflammatory diseases of nasal mucosa mediated by specific immunoglobulin E (IgE) after the susceptible children are exposed to allergens in the environment [1, 2]. Allergic rhinitis is a very common clinical disease in recent years, the incidence of which is as high as 40% in the general population, and the main clinical characteristics are nasal congestion, rhinitis, repeated sneezing, and runny nose [3]. Due to the puerile organs of children, improper late nursing will cause the weakness of children's lungs and spleen and increase the probability of allergic rhinitis [4]. In addition to individual constitution, heredity, allergen, and environmental changes can lead to allergic rhinitis, which affects the quality of children's lives [5–9].

The Apriori algorithm can obtain strong association rules in products, thereby improving the calculation method of similarity between users and optimizing the recommendation results. The Apriori algorithm can evaluate the user's interest in the product by paying attention to the user's implicit behavior information of the product and the evaluation of other users. Data mining mainly uses specific mining algorithms to search for potential rules or patterns in data. At present, data mining algorithms are used in data classification, clustering, association analysis, trend prediction, outlier analysis, etc. [10]. The key rule algorithm used in data mining can not only realize the classification or association of categories, levels, and dimensions but also evaluate the mining performance of the algorithm from the perspectives of space-time complexity, validity, completeness, interactivity, and visualization [11]. There are many traditional Chinese medicines, and memory is difficult, so searching and searching are extremely important. The use of data mining algorithms can improve the search efficiency and promote the treatment of diseases. There are some popular association rule algorithms such as Apriori algorithm, partition algorithm, frequent pattern growth algorithm, direct hash and pruning algorithm, and Eclat algorithm [12]. Apriori algorithm is an algorithm that has a strong influence on frequent itemsets of association rules and can be used for Boolean, single-level, and one-dimensional data association [13]. Apriori algorithm can improve the efficiency of data mining and work efficiency. This study uses data mining algorithms to analyze the differences in execution time and the number of mining association rules between the classic Apriori algorithm and the improved Apriori algorithm under different support thresholds. The difference of the execution time of the classic Apriori algorithm and the improved Apriori algorithm under different attributes is compared, and the impact of the threshold setting based on interest on the execution time of the algorithm and the number of mining association rules is compared. This work can improve the efficiency of data mining through the Apriori algorithm, understand the laws of traditional Chinese medicine in the treatment of children with allergic rhinitis, and provide new ideas for the clinical treatment of children with allergic rhinitis.

## 2. Methods

### 2.1. The Apriori Data Mining Algorithm

The central idea of the classical Apriori algorithm is firstly finding all frequent itemsets *k* that meet the minimum support and searching the iterated item sets (*k* + 1) layer by layer.

Equation (1) represents the association rule of the itemset if the two item sets are *U* and *Z*.

(1) $$\begin{array}{c} R=U⟶Z\left(U\cap Z\right). \end{array}$$

If the times of occurrences of item set *U* in Equation (1) are expressed as *n*(*U*) and the data set is expressed as *A*, the support *S*(*U*⟶*Z*) can be defined as shown in

(2) $$\begin{array}{c} S\left(U⟶Z\right)=\frac{\left[n\left(U\cap Z\right)\right]}{\left|A\right|}. \end{array}$$

Then, the confidence coefficient *δ*(*U*⟶*Z*) can be defined.

(3) $$\begin{array}{c} \delta \left(U⟶Z\right)=\frac{\left[n\left(U\cap Z\right)\right]}{n\left(U\right)}. \end{array}$$

When the iterative search of data is performed by the Apriori algorithm, the conditions in Equation (4) need to be simultaneously satisfied.

(4) $$\begin{array}{c} \left\{\begin{array}{c} S\left(U⟶Z\right)\geq \sup\_\min,\\ \delta \left(U⟶Z\right)\geq \text{conf}\_\min. \end{array}\right. \end{array}$$

Consequently, the Apriori algorithm has the following characteristics. (I) The threshold set that is greater than the support degree, that is, the frequency of the occurrence of targets in the frequent itemset *k* needs to be greater than the minimum support degree. (II) A target with a length less than *k* does not contain any frequent itemset *k*. (III) When itemset *k* − 1 is used to search item set *k*, the automatic link of *k* − 2 of different itemsets can obtain overactive itemset or infrequent itemset.  Figure 1 shows the basic flow of the Apriori algorithm.

### 2.2. The Improved Apriori Data Mining Algorithm

The traditional Apriori algorithm obtained all frequent itemsets. Association mining of potential rules in big data was performed by setting a minimum confidence threshold. The Apriori algorithm was improved by introducing the degree of interest for the mining demand of medical big data. In Equation (5), the model of interest degree was defined.

(5) $$\begin{array}{c} \text{Int}\left(U⟹Z\right)=\delta \left(U⟹Z\right)-\delta \left(\bar{U}⟹Z\right). \end{array}$$

In Equation (5), *δ*(*U*⟹*Z*) was the confidence of the association rule (*U*⟹*Z*) and represented the occurrence rate of the latter item *Z* when the former item *U* appeared. $\delta \left(\bar{U}⟹Z\right)$ was the confidence of association rule $\left(\bar{U}⟹Z\right)$ and represented the occurrence rate of the latter item *Z* when the former item *U* did not appear.

When the Apriori algorithm was improved by using interest degree, in addition to the minimum confidence threshold *δ*_min_, the threshold Int_min_ of the minimum degree of interest was set initially. Then, the association rules of interest were output. Equation (5) shows the calculation of the interest degree.

To verify the performance of the improved algorithm for data association, the classical Apriori algorithm and the improved Apriori algorithm were simulated. The data mining sets were used to simulate the algorithm. Simulation requirements included Intel Core i5 CPU 3.20 GHz, 4 GB memory, Windows 10 operating system, and JAVA language to write algorithms.

### 2.3. Information Sources and Standardized Processing

The *Dictionary of Traditional Chinese Medicine Formulae* was used as the basic information source of traditional Chinese medicine formulae, and the selection of traditional Chinese medicine formulae was performed by referring to *The Chinese Medical Code* and *Traditional Formulae*. The requirements were as follows. (I) The efficacy of rhinitis syndrome was described, including “relieving stuffy nose” and “stopping the runny nose”; (II) Chinese medicinal prescriptions were widely used in the treatment of the main symptoms of rhinitis, such as nasal obstruction, “Bi-Qiu,” and “Bi-Yuan”; (III) Chinese medicine prescriptions had complete information, such as prescription name, drug composition, therapeutic efficacy, and direction of indication.

*The Pharmacopeia of the People's Republic of China*, *Chinese Materia Medica*, *Dictionary of Traditional Chinese Medicine*, and *Traditional Chinese Medicine* were used to standardize the names of traditional Chinese medicines. For example, Fa Ban Xia, Qing Ban Xia, and Zhi Ban Xia were all standardized as Pinellia Ternata.

The standardized treatment of allergic rhinitis syndrome type was implemented by referring to *The Basic Theory of Traditional Chinese Medicine* and *Diagnosis of Traditional Chinese Medicine*. For instance, the “lung and spleen-Qi deficiency” and “Qi deficiency of both lung and spleen” were standardized as “lung and spleen-Qi deficiency.” The “lack of healthy Qi,” “unstable healthy Qi,” and “chronic illness and body deficiency” were standardized as the “deficiency of healthy Qi syndrome.” The criteria of “external contraction of wind evil,” “pathogenic wind attacking the superficies,” and “stuffy nasal passage” were standardized as “wind evil invading the lung.”

Data mining of the curative effect of traditional Chinese medicine on allergic rhinitis in children was performed by using the Chinese traditional Medicine database. The Database of Chinese Medicine was established in 1984 by the *Institute of Traditional Chinese Medicine Information*, *China Academy of Chinese Medical Sciences*. It contained 48 databases and more than 1.2 million data pieces. The keywords were retrieved such as “allergic rhinitis”, “rhinitis”, “infantile”, “children”, and “traditional Chinese medicine”, and the data to be needed were extracted from the literature.

### 2.4. Data Analysis

Frequency analysis was used to analyze the composition of drugs commonly used in the traditional Chinese medicine prescriptions and the meridian and viscera of property and taste of drug composition. The first was frequency number analysis. The frequency of occurrence of traditional Chinese medicine in each traditional Chinese medicine prescription was obtained from top to bottom to reflect the proportion of occurrence of high-frequency drugs in the total drugs. The second was frequent itemset analysis. The set of traditional Chinese medicines in traditional Chinese medicine prescriptions was taken as the itemset, and the frequent itemset was used to mine the common drugs and drug combinations. The fourth was the improved association analysis of the Apriori algorithm. The proportion of the number of prescriptions where there was the cooccurrence of the former and the latter medicine to the total prescriptions was analyzed (support degree). The probability of the occurrence of the latter medicine after the occurrence of the former one was analyzed (confidence degree). The last was curative effect analysis. The changes of clinical symptoms and signs scores of the children with allergic rhinitis before and after the treatment were extracted.

### 2.5. Statistical Analysis

Excel 2016 was employed for the collation of all the extracted data. SPSS 19.0 was employed for statistical analysis of therapeutic effect indexes. The differences among groups were compared by using an independent sample *t*-test. The difference was statistically significant with *P* < 0.05.

## 3. Results

### 3.1. Performance Verification of the Apriori Algorithm before and after Improvement

In Figures 2(a) and 2(b), the execution time of the classical Apriori algorithm and the improved Apriori algorithm and the number of mining association rules decreased with the increase of the support thresholds. The execution time and the number of mining association rules of the improved Apriori algorithm were always smaller than those of the classical Apriori algorithm. In Figure 2(c), the execution time of the classical Apriori algorithm and the improved Apriori algorithm increased with the increase of attribute item numbers. The execution time of the improved Apriori algorithm was always shorter than that of the classical Apriori algorithm.

In Figure 3, with the decrease of the threshold value of interest degree, the execution time of the improved Apriori algorithm and the number of mining association rules gradually decreased. When the threshold value was 0.45, the execution time of the improved Apriori algorithm and the number of mining association rules gradually tended to be stable. Therefore, in the subsequent investigation, the threshold value of the interest degree of 0.45 was selected to improve the Apriori algorithm.

### 3.2. Statistics of Chinese Medicine Treating Allergic Rhinitis in Children

Figure 4 shows the analysis of traditional Chinese medicine and the types of drugs used to treat allergic rhinitis in children. From high frequency to low frequency, the commonly used traditional Chinese medicines for the treatment of allergic rhinitis in children included magnolia (1), cedar (2), Angelica plate (3), Aspergillus flavus (4), Atractylodes macrocephala (5), liquorice (6), Astragalus (7), yellow flower (9), dandelion (10), Asarum (11), savvy (12), menthol (13), plum (14), and Pinellia (15). From high frequency to low frequency, the categories of traditional Chinese medicine for the treatment of allergic rhinitis in children included sweating medicines (1), supplementary medicines (2), heat-clearing and detoxifying medicines (3), phlegm and cough medicines (4), astringent medicines (5), dampness-clearing medicines (6), Qi-regulating medicines (7), wind-expelling and dehumidifying medicines (8), digestive medicines (9), blood circulation-promoting and stasis-dispersing medicines (10), wind-expelling and heat-clearing medicines (11), internal warming medicines (12), sedatives (13), anti-lung-cooling medicines (14), and analgesics (15).

Figure 5 shows the statistics of commonly used prescriptions of traditional Chinese medicine for the treatment of allergic rhinitis in children. The top 20 prescriptions were Jude screen powder, fruit yellow sauce powder, homemade prescription, dental floss magnolia powder, Shenling Baizhu powder, Sijunzi decoction, carminative and Xuanqiao decoction, forsythia powder, rhinitis prescription, Wendan decoction, special achievement powder, Xu's rhinitis prescription, Buzhong Yiqi decoction, Gegen decoction, Guben Tongqiao decoction, Qingxue Qufeng decoction, Qingrui Tongqiao decoction, Erchen decoction, Wenfeijianfei decoction, and Xiaochaihu decoction.

### 3.3. Association Rule Analysis of the Commonly Used Chinese Medicine in Treating Allergic Rhinitis in Children

Figure 6 shows the association rule analysis of commonly used traditional Chinese medicine in the treatment of allergic rhinitis in children. In two-flavor drugs, Perilla frutescens, Saposhnikovia divaricata, ginseng, Notopterygium root, and Astragalus membranaceus were often mixed with liquorice, Flos magnoliae were usually mixed with Fructus xanthii and black plum, and Saposhnikovia divaricata were mixed with Atractylodes macrocephala Koidz (Figure 6(a)). In three-flavor drugs, the confidence degree of Radix angelicae, Astragalus propinquus Schischkin, and Saposhnikovia divaricata was the highest (89.14%), followed by that of liquorice, Saposhnikovia divaricata, and Radix angelicae (87.03%) (Figure 6(b)). The support degree of Radix angelicae, Fructus xanthii, and Atractylodes macrocephala Koidz was the highest (38.23%), followed by that of Astragalus propinquus Schischkin, Saposhnikovia divaricata, and Atractylodes macrocephala Koidz (28.36%) (Figure 6(b)). In four-flavor drugs, the confidence degree of Atractylodes macrocephala Koidz, Radix angelicae, Fructus xanthii, and Saposhnikovia divaricata was the highest (90.85%), followed by that of Saposhnikovia divaricata, Radix angelicae, Flos magnoliae, and Fructus xanthii (84.67%). The support degree of Saposhnikovia divaricata, Radix angelicae, Fructus xanthii, and Flos magnolia was the highest (28.93%), followed by that of Saposhnikovia divaricata, Radix angelicae, Flos magnoliae, and Fructus xanthii (27.81%) (Figure 6(c)).

### 3.4. Curative Effect of Traditional Chinese Medicine on the Treatment of Allergic Rhinitis in Children

Figure 7 shows the efficacy of traditional Chinese medicine in treating allergic rhinitis in children. The results showed that, compared with the signs before treatment, the signs of nasal obstruction, nasal itching, runny nose, sneezing, swelling of the inferior turbinate, and abnormal color of the nasal mucosa in children with allergic rhinitis after the treatment of traditional Chinese medicine compounds were signally reduced (*P* < 0.05).

## 4. Discussion

Glucocorticoids and antihistamines are commonly used in the clinical treatment of allergic rhinitis in children, but most of them can only relieve the clinical symptoms of children, and the recurrence rate and adverse reaction rate are high [5, 14]. Compared with western medicine treatment, traditional Chinese medicine treatment has fewer side effects and less damage to the body and can fundamentally remove the cause of the disease, improve the condition more thoroughly, and prevent recurrence. Traditional Chinese medicine is widely used in the elderly and children, and chronic diseases are often treated with traditional Chinese medicine. According to traditional Chinese medicine, for pediatric allergy, the conditioning of lung and spleen function needs to be emphasized. Besides, consolidating and cultivating fundamental vitality are the foundation of adjusting the balance of Yin and Yang [15]. The nose is the outer phenology of the lung, and the outer phenology reflects the inner. Consequently, regulating the lung and unblocking stuffy nose is the truth of the treatment of this disease. Currently, traditional Chinese medicine has certain advantages in the treatment of allergic rhinitis in children, and it can improve the long-term efficacy of the disease, which is proved [16–18]. However, there are great differences in the understanding of the etiology and pathogenesis of the disease among traditional Chinese medicine experts, and the thinking of medication is also different, so the principles of treatment are not unified. Hence, the data mining method was used to explore the law and efficacy of Chinese medicine prescription in the treatment of allergic rhinitis in children.

The Apriori algorithm is a kind of data mining algorithm that is often used for association rule analysis. Nevertheless, the adoption of the Apriori algorithm to medical big data mining has the following limitations [13, 19]. Firstly, the result error of the strong association rule is large and inconsistent with the actual situation, so it will lead to misdirection. Secondly, the Apriori algorithm can only determine the association rules by setting support *S* and confidence *δ* thresholds. If the threshold is set too much high, the complexity of the algorithm is increased. If the threshold is set too much low, the integrity of the algorithm cannot be guaranteed. Thirdly, when the Apriori algorithm generates the candidate frequent itemset, it needs to browse all the databases. If the database is huge, the load of the system will be increased as well as the complexity of the algorithm. Therefore, the model of interest degree was introduced to improve the Apriori algorithm. Through the simulation test, the execution time of the improved Apriori algorithm was observably reduced, which indicated that the introduction of the interest-based model helped improve the running speed of the Apriori algorithm. Furthermore, the number of attribute items of the improved Apriori algorithm was smaller than that of the classical Apriori algorithm, which indicated that the introduction of the interest degree model was helpful to reduce the redundancy and space occupancy of the algorithm based on the guarantee of the accuracy and stability of the Apriori algorithm [20].

According to the analysis of the medication rule of Chinese medicine compounds in the treatment of allergic rhinitis in children, the compound with the highest frequency was Yu Ping Feng powder, a famous prescription for invigorating the spleen for benefiting lung, and it was used for the treatment of lung diseases such as lung and spleen deficiency and cold wind invading the lung [21]. Through the high-frequency drug analysis, the first 5 commonly used drugs were Flos magnoliae, Saposhnikovia divaricata, Radix angelicae, Fructus xanthii, and Atractylodes macrocephala Koidz. The efficacy of Flos magnoliae was on the lung and stomach, which could disperse cold and unblock the stuffy nose. The efficacy of Saposhnikovia divaricata was on the bladder, lung, spleen, and liver, which could dispel wind, relieve the heat, clear dampness, and relieve pain. The efficacy of Radix angelicae was on the lung, stomach, and intestine, which could dispel wind, clear dampness, tongqiao, and relieve pain. The efficacy of Fructus xanthii was on the lung, which could dispel wind, clear dampness, and relieve the stuffy nose. The efficacy of Atractylodes macrocephala Koidz was on the spleen and stomach, which could invigorate the spleen, supplement Qi, clear dampness, and promote urination. In traditional Chinese medicine, allergic rhinitis was closely related to the evil of cold wind, and the main internal cause of the disease was the deficiency of the spleen and lung. Consequently, both internal therapy and external therapy were considered, and the treatment of both manifestation and root cause was necessary [8]. The main dialectical points of allergic rhinitis were episodic rhinitis, continuous sneezing, runny nose, nasal congestion, and cough [22]. The effects of traditional Chinese medicine on allergic rhinitis in children were evaluated regarding the sign score's abnormal changes of nasal obstruction, nasal itching, runny nose, sneezing, swelling of the inferior turbinate, and abnormal color of the nasal mucosa. The results showed that after the treatment, the signs of nasal obstruction, nasal itching, runny nose, sneezing, swelling of the inferior turbinate, and abnormal color of the nasal mucosa were evidently reduced. Therefore, the treatment of traditional Chinese medicine treatment on allergic rhinitis in children had excellent clinical efficacy, which helped relieve the symptoms of children.

## 5. Conclusion

The model of interest degree was introduced to improve the Apriori algorithm, which can not only ensure the accuracy and stability of the algorithm association mining but also improve the running efficiency of the algorithm and reduce the redundancy and space occupancy of the algorithm. The drug categories of Chinese medicine compounds in treating children with allergic rhinitis were rich. In addition to the treatment of the main pathogenesis of the disease, traditional Chinese medicine also included the treatment of pathological products. The database was only used to analyze the treatment of allergic rhinitis in children with traditional Chinese medicine. Only the index of the sign score was enrolled for the efficacy evaluation, and the efficacy evaluation of other traditional Chinese medicine methods was not analyzed, such as acupuncture, moxibustion, and acupoint application. In the future, it will be combined with clinical research to comprehensively analyze the efficacy of traditional Chinese medicine in the treatment of allergic rhinitis in children. The results of the investigation can provide a reference for the choice of the treatment of traditional Chinese medicine for allergic rhinitis in children.

## Figures and Tables

**Figure 1:** The basic flow of the Apriori algorithm.

**Figure 2:** Performance analysis of the classical Apriori algorithm and the improved Apriori algorithm under different support thresholds and attribute item numbers. (a) Effect of support threshold on the execution time of algorithms; (b) effect of support threshold on the number of association rules mined by algorithms; (c) effect of attribute item numbers on the execution time of algorithms.

**Figure 3:** Performance analysis of the improved Apriori algorithm under different thresholds of interest degree. (a) Effect of the threshold of interest degree on the execution time of algorithms; (b) effect of the threshold of interest degree on the number of association rules mined by algorithms.

**Figure 4:** Analysis of traditional Chinese medicine and drug types of the treatment of allergic rhinitis in children. (a) The top 15 high-frequency Chinese medicines, namely, Flos magnoliae, Saposhnikovia divaricata, Radix angelicae, Fructus xanthii, Atractylodes macrocephala Koidz, liquorice, Astragalus propinquus Schischkin, Poria cocos, Ephedra, dandelion, Asarum, Semen cassiae, menthol, plum, and Pinellia ternate. (b) The top 15 categories of traditional Chinese medicines, namely, diaphoretic drug, restoring deficiency drug, heat-clearing and detoxicating drug, drug of eliminating phlegm and stopping cough, astringent, damp-clearing drug, Qi-regulating drug, medicine for removing pathogenic wind and dampness, digestant drug, medicine for promoting blood circulation and dispersing blood stasis, medicine for dispelling wind and clearing heat, interior-warming drug, tranquilizer, medicine for clearing away the lung heat and dissipating heat, and Tongqiao and analgesic medicine.

**Figure 5:** Statistics of the commonly used prescriptions of traditional Chinese medicine for the treatment of allergic rhinitis in children. 1-20 on the *x*-axis: Jude screen powder, Fructus xanthii powder, self-made prescription, Flos magnolia powder, Shenling Baizhu powder, Sijunzi decoction, dispelling wind and Xuanqiao decoction, forsythia powder, prescription for rhinitis, Wendan decoction, special achievement powder, Xu's rhinitis prescription, Buzhong Yiqi decoction, Puerariae decoction, Guben Tongqiao decoction, Qingxue Qufeng Decoction, Qingrui Tongqiao decoction, Erchen decoction, Wenfeijianfei decoction, and Xiaochaihu decoction.

**Figure 6:** Association rule analysis of Chinese medicine prescription for the treatment of allergic rhinitis in children: (a) analysis among the one-flavor drugs; (b) analysis of the two-flavor drugs versus the one-flavor ones; (c) analysis of the three-flavor drugs versus the one-flavor ones.

**Figure 7:** Comparison of the sign scores of children with allergic rhinitis before and after treatment. 1-6: nasal obstruction, nasal itching, runny nose, sneezing, swelling of the inferior turbinate, and abnormal color of the nasal mucosa. ∗ meant that compared with the sign scores before the treatment, *P* < 0.05.

## Data Availability

The data used to support the findings of this study are available from the corresponding author upon request.

## References

[1] Schuler Iv C. F., Montejo J. M. (2019). Allergic rhinitis in children and adolescents. *Pediatric Clinics of North America*.

[2] Brown T. (2019). Diagnosis and management of allergic rhinitis in children. *Pediatric Annals*.

[3] Tajima H., Pawankar R. (2019). Obesity and adiposity indicators in asthma and allergic rhinitis in children. *Current Opinion in Allergy and Clinical Immunology*.

[4] Norhafizah S., Salina H., Goh B. S. (2020). Prevalence of allergic rhinitis in children with otitis media with effusion. *European Annals of Allergy and Clinical Immunology*.

[5] Prieto A., Rondón C., Eguiluz-Gracia I. (2021). Systematic evaluation of allergic phenotypes of rhinitis in children and adolescents. *Pediatric Allergy and Immunology*.

[6] Nieto A., Nieto M., Mazón Á. (2021). The clinical evidence of second-generation H1-antihistamines in the treatment of allergic rhinitis and urticaria in children over 2 years with a special focus on rupatadine. *Expert Opinion on Pharmacotherapy*.

[7] Mener D. J., Lin S. Y. (2015). Improvement and prevention of asthma with concomitant treatment of allergic rhinitis and allergen-specific therapy. *International Forum of Allergy & Rhinology*.

[8] Feng L., Lin L., Wang S. (2021). Clinical practice guidelines for the treatment of allergic rhinitis in children with traditional Chinese medicine. *The Anatomical Record*.

[9] Liang J., Gu Q. (2021). Current status of Chinese herbal medicine to treat allergic rhinitis in children: from the perspective of Western medicine-a narrative review. *Translational Pediatrics*.

[10] Mellor J. C., Stone M. A., Keane J. (2018). Application of data mining to “big data” acquired in audiology: principles and potential. *Trends in Hearing*.

[11] Ryu S., Song T. M. (2014). Big data analysis in healthcare. *Healthcare Informatics Research*.

[12] Li Q., Zhang Y., Kang H., Xin Y., Shi C. (2017). Mining association rules between stroke risk factors based on the Apriori algorithm. *Technology and Health Care*.

[13] Zheng Y., Chen P., Chen B., Wei D., Wang M. (2021). Application of Apriori improvement algorithm in asthma case data mining. *Journal of Healthcare Engineering*.

[14] Đurić-Filipović I., Caminati M., Kostić G., Filipović Đ., Živković Z. (2016). Allergen specific sublingual immunotherapy in children with asthma and allergic rhinitis. *World Journal of Pediatrics*.

[15] Yen H. R., Liang K. L., Huang T. P., Fan J. Y., Chang T. T., Sun M. F. (2015). Characteristics of traditional Chinese medicine use for children with allergic rhinitis: a nationwide population-based study. *International Journal of Pediatric Otorhinolaryngology*.

[16] Huang S. K., Ho Y. L., Chang Y. S. (2015). Prescriptions of traditional Chinese medicine, Western medicine, and integrated Chinese-Western medicine for allergic rhinitis under the National Health Insurance in Taiwan. *Journal of Ethnopharmacology*.

[17] He S., Li Y., Chen J. (2014). Integrated traditional Chinese and Western medicine clinical research for the treatment of allergic rhinitis in children. *Journal of Clinical Otorhinolaryngology, Head, and Neck Surgery*.

[18] Guo H., Liu M. P. (2013). Mechanism of traditional Chinese medicine in the treatment of allergic rhinitis. *Chinese Medical Journal*.

[19] Lu P. H., Keng J. L., Kuo K. L., Wang Y. F., Tai Y. C., Kuo C. Y. (2020). An Apriori algorithm-based association rule analysis to identify herb combinations for treating uremic pruritus using Chinese herbal bath therapy. *Evidence-based Complementary and Alternative Medicine*.

[20] Ou J., Zhang J. (2022). Data mining and meta-analysis of psoriasis based on association rules. *Journal of Healthcare Engineering*.

[21] Chan H. H. L., Ng T. (2020). Traditional Chinese medicine (TCM) and allergic diseases. *Current Allergy and Asthma Reports*.

[22] Fu Y., Kong Y., Li J. (2020). Mesenchymal stem cells combined with traditional Chinese medicine (qi-fang-bi-min-tang) alleviates rodent allergic rhinitis. *Journal of Cellular Biochemistry*.

